This article has been retracted.

# Higher Education Environment Monitoring and Quality Assessment Model Using Big Data Analysis and Deep Learning

**DOI:** 10.1155/2022/7281278

**Published:** 2022-10-05

**Authors:** Hanfei Wu

**Affiliations:** Department of Humanities and Social Sciences, Nantong University, Nantong 226019, China

## Abstract

A university exists to help students develop their skills. The goal of university development is to raise the standard of personnel training, and the core component of university development is teaching quality. Whether the level of practical training can as soon meet the requirements of enterprise employment. For responding to the demands of professions and occupations, it is essential. Teaching quality evaluation is a crucial cornerstone for ensuring the quality of instruction. Universities and colleges should therefore concentrate on evaluating instruction. Schools and colleges can more rapidly and thoroughly comprehend how their off-campus cooperative adult education programmes are running while also enhancing the efficacy and impartiality of their quality assessment by utilising educational data mining and learning analysis technology. Currently, issues with backward evaluation instruments, a single evaluation topic, and easy evaluation methods exist when evaluating the quality of schooling. Big data technology is used to create a higher vocational education environment monitoring and quality evaluation system that offers new and varied approaches to evaluate teaching quality. The technique for evaluating the quality of schooling is expanded upon in this research using various big data mining technologies. The improved collaborative filtering algorithm's mean absolute difference is approximately 18.23% when the data set is larger. In conclusion, when applied to big data sets, the technique in this work performs with greater accuracy than the conventional collaborative filtering algorithm. The scoring matrix becomes denser as there are more scoring items in the model. In turn, this results in a more accurate similarity calculation at the beginning of the programme, albeit the similarity calculation error increases as the scoring matrix becomes denser.

## 1. Introduction

The core of higher education quality is teaching quality. The concept of higher education quality has a direct impact on the formation of the concept of teaching quality. Its multilevel nature makes teaching quality have diversified understanding [1]. Teaching quality is the overall structure of talent training specifications, is a system formed by continuous development, is the overall result of school running and teaching management, and is a complex dynamic process and improvement. Improving teaching quality is to strengthen the quality of talent practice, that is, to train students to have good basic knowledge structure, solid professional knowledge and skills, strong practice and innovation ability, and good psychological and physical quality [2]. Use modern educational technology to truly and comprehensively collect, mine, and analyze big data, explore the direction, path, and method of acquiring dynamic information on teaching and learning, and dynamically grasp student learning paths, teachers' teaching paths, and school teaching management strategies [3]. Compared with traditional data, big data has the features of unstructured, distributed, mass quantity, data analysis has changed from expert level to user level, and visual display is widely used. There is a need for the establishment of a basic higher education quality model [4].

In order to conduct an all-encompassing and multifaceted inspection and assessment of education, a strong education quality evaluation system should be built on broad support and involvement and utilise a variety of evaluation subjects [5]. In order to encourage teachers and students to consciously commit themselves to educational reform and increase the enthusiasm of education quality, the fundamental goal of education quality evaluation in universities is not to reward and punish or grade, but rather to form a scientific and reasonable incentive mechanism through evaluation and form a fair and benign competition environment [6]. The system for evaluating the quality of education should take into account both static, simple-to-use, and easy-to-describe educational parameters as well as dynamic, complex-to-use, and hard-to-quantify indications produced by the interplay of numerous components. In order to improve the indicators of teaching quality evaluation in higher education, this article analyzes and studies the fundamental state data of teaching in universities, explores new methods and new methods of teaching quality monitoring, examines the key determinants of teaching quality, and builds a teaching quality monitoring data model. Facilitate the extraction and analysis of different types of text data. To more completely and precisely reflect the issues in the actual teaching process, both qualitative and quantitative methodologies are applied during the analytic phase.

Digital campuses and informatization of education and teaching have become the main challenges facing higher education today [7]. A lot of data is continually being produced by students, teachers, administrators, instructional processes, learning approaches, etc. [8]. The regular and valuable information contained in these big data cannot, however, be used to turn material resources into good accounts for their effectiveness because the traditional system for evaluating teaching quality is unable to integrate and sort out these teaching big data in a timely and efficient manner. The thorough assessment of educational quality is based on large data from numerous sources. Planning, storing, and using big data responsibly have become crucial to development and reform. On the one hand, utilising information technology to enhance the process of evaluating educational quality can lighten the workload. On the other hand, implementing universal criteria for evaluation can increase evaluation accuracy to some extent [9].

Through big data mining, students' learning feedback information should be objective and credible. They can use this feedback information to improve and improve their own education methods, better set up courses, adjust teaching contents and teaching plans according to students' learning results, and improve teaching effects through these methods. The innovation of this article lies in the following: (1) The data set for the education quality study is further optimised using the deep learning-based quality evaluation model. Currently, only routine records and data are collected, and the data collection is also based on energy data. The next stage is to increase text data collecting and analysis based on the data already available and work to more accurately reflect the current state of education quality. (2) Combined with big data mining technology [10], the education quality monitoring model is improved. Constantly revise the core indicators of education quality, and improve the weight of each indicator through more sample data. At the same time, it studies the methods of special monitoring for specific aspects and continuously introduces various monitoring results, striving to realize intelligent education quality monitoring, intelligent education quality evaluation, and intelligent education decision-making.

## 2. Related Work

The primary content and fundamental structure of teaching assessment, according to Pennie I's proposal, are the effective use of big data in the routine monitoring of teaching status data. The fundamental status of teaching in universities is mirrored by data, and data analysis aids schools [11], in accordance with the internal regulations of teaching work and Internet big data technology. Veronica et al. believe that the structural level of the current higher education system is characterized by diversification and complexity. The education system is progressive from each link to the next, and there are many influencing factors. Therefore, the quality of the guidance system is very important to the higher education system [12]. The education evaluation system studied by Chen Q not only has the function of evaluating the level of students, teachers, and universities but also has the function of testing the educational reform achievements of universities, providing a good basis for improving the education system and promoting the vigorous development of the education theory system [13]. According to Megnounif et al., for the students themselves, the system can assist in the management of comprehensive quality evaluation related materials; more importantly, it can enable students to fully understand their comprehensive quality level, help them plan their own development direction and path, make up for defects, and promote students to improve their comprehensive quality level from their own perspective [14]. Shauchenka and Buslowska further pointed out that when evaluating the level and benefit of running a school, it should be classified and evaluated according to the nature of colleges and departments and systems. And similar schools should also make hierarchical evaluation according to different situations, so that the evaluation scheme formulated in this way is more feasible [15]. According to the analysis of Shengquan and Xiaoqing, it is necessary to have a scientific evaluation method and feedback the evaluation results to the teachers to guide the teaching reform direction. It is of great significance to improve the quality of practical teaching and cultivate the characteristics of practical teaching [16]. The teaching quality assessment management information system constructed by Bebenina has a certain degree of openness, making the data interface flexible and transmitting data with other information systems, such as basic information of students, basic information of teachers, and basic information of educational affairs, to achieve information sharing. The system uses user-defined settings for evaluation forms, evaluation items, evaluation indicators, evaluators, and evaluators. After initialization, an evaluation questionnaire is generated [17]. In the aspect of education big data algorithm, Dai proposed a clustering algorithm based on map/reduce, which achieved obvious results in a variety of performance indicators under the parallel frameworks such as speed growth and scale growth and then gradually formed a collaborative clustering framework under the parallel environment [18]. Patel and Desai focused on the research of association rule algorithm and made some improvements on the classical Apriori algorithm [19]. Li et al. designed the useful mode of distance education platform and network education platform based on Web log mining technology [20].

Research on the use of data mining technology in the field of education is still in its infancy, according to an analysis of pertinent literature from both domestic and foreign sources. Particularly, more research is required on the use of data mining in teaching management, and it will be useful to understand how to use data mining to achieve personalised analysis of teaching data and the creation of education quality systems.

## 3. Application of Big Data Mining and Deep Learning in Educational Evaluation System

The analysis and suggestion features of the system for evaluating teaching quality that was created in this article show how sophisticated the system is. Through this technology, the evaluators can evaluate every teacher online and use the detailed evaluation data to modify each teacher's work. The deep learning algorithm is used to develop the system for evaluating the quality of instruction (as shown in Figure 1). The system created in this way is highly intelligent. According to the issues and weak points in the teaching process, it accurately assesses the teaching quality and makes logical recommendations for teaching improvement. The gathering of teaching big data is the most fundamental component of the big data-based system for evaluating the quality of instruction. The only way to measure and evaluate the teaching quality is to thoroughly gather and screen useful data. We must gather huge data on the entire teaching process and ensure data gathering is normalised in order to successfully develop a new, rational, scientific system for evaluating the quality of instruction.

Mining valuable information for teaching quality evaluation from massive data, classifying and storing, and then forming a comprehensive and scientific teaching quality evaluation analysis report were performed. In the process of evaluating teaching quality, it covers a wide range of evaluation indicators and forms large-scale complex data. Most of the teaching quality evaluation systems can only display the teaching quality of teachers and do not have the ability to intelligently analyze the problems of teachers. However, the research shows that the deep learning algorithm can accurately extract the hidden rules of data and deal with the diversity of complex data. Therefore, the application of deep learning algorithm in the design of teaching quality system is reasonable. By analyzing the evaluation theory of deep learning, the evaluation elements of deep learning are sorted out and summarized, and on this basis, the first level indicators are formed. The index framework is preliminarily drawn up after index refining, divergence, and convergence. Then, solicit relevant experts' opinions and suggestions to revise and improve the indicator framework and finally form a teaching quality evaluation indicator system based on deep learning. The index system construction process is shown in Figure 2.

Analyzing data is a key component of evaluation, which serves as the foundation for evaluating the indicators of education quality. Big data analysis can ensure the accuracy of analysis and judgement, achieve the diversity of the evaluation system, and combine the evaluation with various educational levels (see Figure 3). The empirical technique has been used in higher education evaluation practice. Although this method is quick and convenient, it cannot be fair and objective because it is significantly influenced by the subjective consciousness of managers and evaluators. The establishment of a model for measuring teaching quality using scientific processes and methods is absolutely required. In order to identify the key issues in school-running management and teaching quality, experts and scholars with extensive knowledge and experience in this field visit universities, work closely with higher education management staff, and utilise a variety of scientific approaches. Perform a quantitative or qualitative analysis supported by evidence, pinpoint the root causes of issues, put forth workable improvement plans, and then direct schools in putting the plan into action. The process of value judgement on the school running level, teaching quality, and students' academic achievements of the college is done in accordance with the evaluation criteria, utilising workable evaluation methodologies and tools, through qualitative and quantitative analysis.

In the process of indicator selection, we follow the systematic principle, and there is a logical relationship between the assurance indicators. From top to bottom, it can effectively reflect the comprehensive quality of students and the teaching level of teachers. In addition, the principles of comparability, operability and quantification should be followed, and indicators that are simple, clear, micro, easy to collect, operable, and comparable should be selected to facilitate data collection in the later period. At the same time, the effectiveness of the evaluation can be ensured. Create various assessment application software, accurately mine and analyze the data, and thoroughly and accurately comprehend the facts on the teaching and learning processes followed by students, teachers, and school administrators. The operability should be considered when choosing evaluation indicators and data collection methods. Simple and convenient indicators should be chosen for the evaluation system, and operability and practicability can guarantee the veracity of the evaluation results. Therefore, in order to ensure that the evaluation system can fully reflect the actual situation of education quality, it should be considered from a comprehensive perspective, and the selection of indicators should not be biased, so as to ensure the objectivity of the indicators. Through the theory and methods of education evaluation, we have obtained the classroom teaching evaluation indicators shown in Table 1 and the professional quality evaluation indicators shown in Table 2.

It is typically important to give each assessment indicator a score when designing evaluation indicators in order to simplify calculation and ease quantifying of evaluation outcomes. To assess each indicator's significance, various weights are simultaneously assigned, using the various ratings for each evaluation indication, followed by a weighted computation using the provided weight. A full indicator system must also assign proportional weights to the indications and make clear the significance of each signal in addition to having the ideal structure.

Curriculum quality evaluation and professional quality evaluation are two indispensable and interrelated tasks in college teaching. On the one hand, curriculum quality construction is the premise and foundation, and only when the curriculum construction has reached a certain level or stage can the curriculum evaluation be conducted. On the other hand, curriculum evaluation can promote the improvement of professional quality. Through the evaluation, we can find out the weak links and shortcomings in curriculum quality, improve and overcome them, and construct a benign continuous improvement mechanism of curriculum quality of “construction-evaluation-development-innovation” with the goal of improving curriculum quality. In addition, the realization of professional training goals depends on a reasonable curriculum system, and the professional training goals are finally implemented on the educated through the teaching of teachers. It can be seen that the professional quality directly affects the quality of personnel training and is related to the overall teaching level of universities.

## 4. Algorithm Description

To fix the issue with the current evaluation system's overly basic evaluation procedures. The foundation of more effectively using mass data technology to address this issue is the acquisition of rich and pertinent information data. The constraints of time and space are overcome by this evaluation method. Big data technologies can not only produce accurate evaluations but also help assessors refine their current evaluation techniques. Without physically visiting the classroom, the evaluators can grade the class data from the gathered class videos and big data analysis.

Combine collaborative filtering with Expert System with application based on association rule data mining technology, record each user's service files, browsing hobbies and habits, and then provide learners with a set of teaching resources. From the centralized analysis of the resources, it can be concluded that each learner has an understanding of the learning knowledge points. Substitute the filtered data into the formula to get the learning cost coefficient of each knowledge point. Then, filter out the inappropriate knowledge points and substitute them into the expectation formula to obtain the average learning cost coefficient of the entire course. The formula is as follows:

(1) $$\begin{array}{c} f=\left(1-\frac{M}{N}\right)\times f_{1}-\left|EP-P\right|\times f_{2}. \end{array}$$

Among them, *f*_1_ is the weight of the distribution of knowledge points, and *f*_2_ is the weight of the difficulty coefficient. When *f*_1_ = 0, it means that only the difficulty coefficient of the test questions is limited, and when *f*_2_ = 0, it means that only the distribution of knowledge points is limited.

A vector model is established to represent the attribute features and the weights of the features, and then, the vector distance is calculated to analyze the similarity of the items. A distance algorithm is mainly divided into similarity calculation based on Euclidean distance and similarity calculation based on cosine. The formula is as follows:

(2) $$\begin{array}{c} dst\left(P_{i},P_{j}\right)=\sqrt{\overset{k=n}{\underset{k=1}{\sum }}{\left(x_{k}-y_{k}\right)}^{2}}, \end{array}$$

where *P*_*i*_, *P*_*j*_ is an *n*-dimensional vector and *x*_*k*_, *y*_*k*_ is the value of the *k*-th dimension of *P*_*i*_, *P*_*j*_, respectively.

Calculate the distance from each object *P* in the data set to the center of cluster *k*:

(3) $$\begin{array}{c} d\left(i,j\right)=\sqrt{\left(x_{1i}-y_{1j}\right)\delta^{2}+}\sqrt{\left(x_{2i}-y_{2j}\right)\delta^{2}}+\cdots +\sqrt{x_{mi}-y_{mj}}. \end{array}$$

Among them, *i*, *j* is two *n*-dimensional data objects.

The user teaching resource matrix serves as the foundation for this algorithm's determination of item similarity. The educational materials that are similar to one another on this basis are grouped, and a comparison between the clustering centers of each category and the item is made. This can significantly narrow the range of searchable things and increase the algorithm's effectiveness. The square error criterion seeks to maximise the similarity of the objects within the cluster in order to maximise the independence and compactness of the clustering findings. Calculate the included angle of cosine to determine how comparable the educational resources are by using the user's understanding of them as an *n*-dimensional vector. The following is the similarity calculation formula:

(4) $$\begin{array}{c} E=\overset{k}{\underset{i=1}{\sum }}{\left|P-m_{i}\right|}^{2}\underset{j=1}{\sum }\xi {\left(m_{j}-1\right)}^{2}. \end{array}$$

Enter *s* teaching resources that need to be classified, recorded as a set:

(5) $$\begin{array}{c} s=\left\{s_{1},s_{2},\cdots ,s_{n}\right\}. \end{array}$$

Enter *m* users as a set:

(6) $$\begin{array}{c} R=\left\{r_{1},r_{2},\cdots ,r_{m}\right\}. \end{array}$$

Because of the large amount of teaching resources data, the calculation of finding adjacent teaching resources in the whole teaching resources space is huge and inefficient. From the nature of clusters, most of the nearest neighbors of the target teaching resources are in the clusters with the highest similarity. Therefore, it is only necessary to find the nearest neighbor clusters of the target teaching resources and then find the nearest neighbor teaching resources from them.

Judgment is a matrix representing the relative importance obtained by comparing the importance of opinion between classes. Relative weight can be obtained by using the judgment matrix-vector weight calculation methods mainly include root sum, root, and logarithmic method of least squares. The method of calculation is as follows:

(7) $$\begin{array}{c} C_{ij}=\frac{\sum_{1}^{m}n_{ik}}{\sum_{i}^{n}n_{jk}}\varphi \left(m_{i}n_{j}\right). \end{array}$$

Since the cooccurrence matrix cannot be read into the memory at one time under the condition of big data, the formula needs to be processed. Let the cooccurrence matrix be

(8) $$\begin{array}{c} \left\{\begin{array}{c} n_{1},n_{2},\cdots ,n_{m},\\ n_{i1},n_{i2},\cdots ,n_{im}. \end{array}\right. \end{array}$$

Then,

(9) $$\begin{array}{c} C_{i}=n_{ij}\varphi_{k}\underset{i=1}{\sum }m_{i}n_{j}. \end{array}$$

However, considering that the cooccurrence matrix must be a symmetric matrix, that is, the number of occurrences of item *i*, *j* is equal to the number of occurrences of item *m*, *n*; the vector can be directly used for calculation. In this way, when calculating the predicted score value *C*_*ij*_, one multidimensional vector can be read in each time instead of the entire matrix.

The transaction data is converted into a two-dimensional compressed Boolean matrix format. Each row of the converted data matrix represents a transaction, and each column represents a group of transaction elements. The same transaction is stored only once in a matrix, and a matrix is created to store the number of iterations of the transaction to achieve the compression of transaction data. Calculate the support of each component according to formula (10), and screen the components that exceed the minimum support.

(10) $$\begin{array}{c} QH=\overset{t}{\underset{n=0}{\sum }}x_{i}\theta_{i}. \end{array}$$

Among them, *x*_*i*_ is each data item, and *θ*_*i*_ is the weight ratio of each data item.

During data cleaning, correcting or clearing data that does not meet the cleaning rules is the first step in quality monitoring. Then, on the basis of monitoring data, the indicators and contents of teaching quality monitoring can be studied, and a higher education quality monitoring model can be constructed.

## 5. Investigation Analysis and Experiment

The teaching process is directly related to multiple data in teaching input and learning output. On the basis of careful analysis of the characteristics of teaching itself and existing data, according to the “input-output” principle, referring to different teaching evaluation indicators and according to the “teaching input-teaching process-learning results” model, the elements of teaching evaluation are determined. The data closely related to teaching quality is the basic index of teaching quality. This method can systematize and quantify the design idea and judgment process and can avoid a large number of uncertain factors. This measure greatly simplifies the calculation work, and it is convenient to unify the design and judgment process in the development process. Therefore, here, the data of a university is chosen as the research project. According to the monitoring index of higher education teaching quality, we can see the situation of each monitoring point by observing the changes of the monitoring index, as shown in Figure 4.

Students, teachers, and experts enter the system to evaluate the corresponding teaching quality index scores. The system management personnel must be able to control whether some personnel can evaluate and query the real-time progress of evaluation on any batch. The effectiveness of the questionnaire of the personnel participating in the evaluation shall be dynamically monitored, and the personnel evaluation process shall be centrally set. Big data can ensure the objectivity of evaluation results. Big data can ensure the objectivity of the evaluation results, because big data can effectively improve the accuracy and reliability of data analysis, and effectively avoid the contingency caused by random sampling of data, so that the data analysis results are more convincing.

Figure 5 shows that the teaching quality evaluation statistics of different subjects show that the model established by this algorithm can identify the relative score comparison of teaching quality evaluation of different courses, and provide different types of data for comprehensive analysis of teaching quality.

The main goals of this study are to gain a thorough understanding of the current state of teaching effect evaluation in higher education, investigate any issues that may arise in this situation through questionnaires, identify the variables influencing students' deep learning, and identify a practical foundation for the design of a deep learning classroom in order to enhance students' capacity for deep learning. The majority of the unified course evaluation systems that are utilised in a daily instruction are “learning from the existing unified course evaluation system.” Online surveys are made available. 200 surveys were disseminated online with the aid of family, friends, teachers, and classmates; 158 of those questionnaires were later found. After invalid questions were eliminated, 123 valid questionnaires remained, yielding a 94% effective questionnaire recovery rate that served as the foundation for subsequent data statistics. All questionnaire data were entered into SPSS25.0 data analysis software for analysis (as shown in Figure 6).

Based on the traditional collaborative filtering algorithm, the idea of clustering algorithm is introduced to narrow the range of similarity and implement the map/reduce strategy on the big data platform. From the characteristics of cooccurrence matrix and online education data, an improved parallel collaborative filtering algorithm is realized. In this article, different big data mining algorithms are introduced into the education quality evaluation system. The average absolute difference of the improved collaborative filtering algorithm is about 18.23% in the case of large data sets. Integrate and merge the data from various subdatabases (teacher management database, teaching database, student learning database, teaching management database, etc.) into a single education theme database, and adjust the data difference to ensure that the original data is consistent with the input standard. A preliminary analysis of the sorted data is carried out, and Figure 7 is obtained.

Most teachers think that the quality of education needs to have its own independent teaching effect evaluation system, and this system needs to be able to comprehensively evaluate the ability of students. In the survey, it was also found that due to the influence of age, education background, professional knowledge, emphasis on the evaluation system, and other factors, only a small number of teachers are very familiar with deep learning. However, based on the fact that the evaluation system can cultivate students' innovative ability, critical thinking ability, hands-on operation ability, and teamwork ability, the vast majority of teachers believe that the evaluation system can cultivate students' deep learning ability, thereby analyzing the effect of evaluation index selection on education quality (as shown in Figure 8).

From the point of view of total quality management, the evaluation of teaching course includes several basic links such as course preparation, teaching process, and after-school arrangement, mainly from the setting of teaching objectives, the arrangement of teaching contents, the design of teaching structure, the choices of teaching ways, and the embodiment of teachers' teaching ability. Therefore, it is very necessary to construct a teaching effect evaluation system which can comprehensively evaluate students' deep learning ability, and it can also promote the classroom to meet the standard requirements and realize the effective teaching feedback of the evaluation system.

Transmission, analysis, and sharing of information and data enable real-time monitoring of the current quality of national education. Teachers, students, parents, and education departments at all levels must all work together and support the creation of a thorough and open platform for education quality evaluation services. As information technology develops, the comprehensive platform for evaluating educational quality will surely become more significant, acting as a catalyst for significant changes in education.

## 6. Conclusion

The weight of the evaluation index is an important part of the teaching index system and cannot be subjective. Therefore, it is necessary to clarify the evaluation object and evaluation content and to pass scientific demonstration. The content of the evaluation index system should be combined with various factors. Big data can realize the accurate positioning of teaching and help the development of talents. The accuracy of this algorithm in large data sets is higher than that of traditional collaborative filtering algorithms. The more scoring items in the model, the denser the scoring matrix. The denser the scoring matrix, the more accurate the similarity calculation will be at the beginning of the programme but the greater the similarity calculation error. Education quality assessment contains a large amount of data. In the actual evaluation, the use of massive data can effectively mine the intrinsic value of massive data and the data content in related fields, thus effectively improving the effect of teaching quality evaluation, using data mining technology to provide a variety of data content for teaching research, so that the teaching results can better adapt to the current teaching reform.

## Figures and Tables

**Figure 1:** Architecture of teaching quality evaluation system based on big data mining.

**Figure 2:** Teaching quality evaluation index system based on deep learning.

**Figure 3:** Teaching quality evaluation index system.

**Figure 4:** Changes in the monitoring index of education and teaching in universities.

**Figure 5:** Evaluation scores of education quality in different disciplines.

**Figure 6:** Evaluation of the teaching situation of different knowledge points.

**Figure 7:** Analysis of the application of the evaluation system.

**Figure 8:** The effect of the selection of evaluation indicators on the quality of education.

**Table 1:** Description of classroom teaching quality indicators.

Number	Indicator content	Score
Q1	Content proficient	0.54
Q2	Strict management	0.42
Q3	Teaching enrichment	0.73
Q4	Inspire innovation	0.65
Q5	Good teaching atmosphere	0.8
Q6	Learn and earn	0.73
Q7	Well organized	0.71
Q8	Smooth expression	0.5
Q9	Innovative teaching techniques	0.72
Q10	Emphasize practical ability	0.62

**Table 2:** Professional quality evaluation indicators.

First-level indicator	Secondary indicator	Three-level indicator
Professional comprehensive quality	Teaching conditions	Faculty (0.56)
		Teaching hardware (0.28)
		Training conditions (0.64)
	Teaching management and implementation	Teaching plan (0.43)
		Curriculum construction (0.87)
		Teaching management (0.68)
	Teaching quality	Professional theory (0.46)
		Employment (0.71)
		Social evaluation (0.56)

## Data Availability

The data used to support the findings of this study are available from the corresponding author upon request.
